The article "A phase II study of the combination chemotherapy of bevacizumab and gemcitabine in women with platinum-resistant recurrent epithelial ovarian, primary peritoneal, or fallopian tube cancer" was published in 2020. Journal: J Ovarian Res.

# A phase II study of the combination chemotherapy of bevacizumab and gemcitabine in women with platinum-resistant recurrent epithelial ovarian, primary peritoneal, or fallopian tube cancer

**DOI:** 10.1186/s13048-020-0617-y

**Published:** 2020-02-07

**Authors:** Shoji Nagao, Ai Kogiku, Kazuhiro Suzuki, Takashi Shibutani, Kasumi Yamamoto, Tomoatsu Jimi, Miho Kitai, Takaya Shiozaki, Kazuko Matsuoka, Satoshi Yamaguchi

**Affiliations:** 1 Department of Gynecologic Oncology, Hyogo Cancer Center, 13-70 Kitaoji-cho, Akashi-city, Hyogo 673-8558 Japan; 2 Department of Obstetrics and Gynecology, Nishi Kobe Medical Center, 5-7-7-1 Kojidai, Kobe-city, Nishi-ku 651-2273 Japan

**Keywords:** Platinum-resistant, Recurrent ovarian cancer, Gemcitabine, Carboplatin

## Abstract

**Introduction:**

Bevacizumab and gemcitabine are key drugs for treating recurrent epithelial ovarian cancer. However, information about the combination of bevacizumab and gemcitabine is insufficient. We conducted a phase II study to assess the feasibility, clinical activity, and toxicity of this combination chemotherapy.

**Methods:**

This study included women with platinum-resistant recurrent epithelial ovarian, primary peritoneal, or fallopian tube cancer who received one to three regimens of platinum-based chemotherapy between April 1, 2015 and December 31, 2018. The patients received bevacizumab 15 mg/kg intravenously on day 1 and gemcitabine 1000 mg/m^2^ intravenously on days 1 and 8 every 21 days until disease progression or unacceptable toxicity. The primary endpoint was the completion rate of three cycles of chemotherapy. This study was registered in the University Medical Information Network (UMIN) Clinical Trials Registry (UMIN000016619).

**Results:**

Among the 19 patients, 18 (95%) received ≥3 and 9 (47%) received ≥6 cycles of the study therapy. The objective response rate was 42% (complete response of 16% and partial response of 26%), and the clinical control rate was 84%. Hematological toxicity included neutropenia grade 3/4 in 9 patients (47%), anemia grade 3/4 in 2 (11%), and thrombocytopenia grade 3/4 in 1 (5%). One patient (5%) had grade 3 hypertension, and 1 (5%) had grade 3 protein urea. Possibly related grade 3 pulmonary toxicity was observed in 1 patient. Three patients needed dose reduction of gemcitabine to 800 mg/m^2^ due to treatment delay by 15 to 21 days on day1. There was no treatment delay more than 14 days on day 8. The median progression-free survival duration was 5.1 months and median overall survival duration was 21.3 months.

**Conclusion:**

The combination chemotherapy with gemcitabine and bevacizumab was feasible, effective and safe. This combination chemotherapy may be explored in a further randomized trial.

The article "A phase II study of the combination chemotherapy of bevacizumab and gemcitabine in women with platinum-resistant recurrent epithelial ovarian, primary peritoneal, or fallopian tube cancer" was published in 2020. Journal: J Ovarian Res.

## Introduction

In the AURELIA trial, the addition of bevacizumab to single-agent chemotherapy significantly improved the response rate (single-agent chemotherapy vs. bevacizumab combination therapy: 11.8% vs. 27.3%, *p* = 0.001) and progression free survival (PFS) duration (median PFS, 3.4 vs. 6.7 months; hazard ratio, 0.48; 95% confidence interval: 0.38 to 0.60, *p* < 0.001) without problematic toxicity in patients with platinum-resistant recurrent ovarian cancer [1]. Based on these findings, bevacizumab combined with single-agent chemotherapy became one of the standard treatments for platinum-resistant recurrent ovarian cancer. However, the AURELIA trial did not include gemcitabine, which is an active agent in patients with recurrent ovarian cancer and appears to be very well tolerated [2, 3].

Gemcitabine is considered as one of the most promising cytotoxic anti-cancer agents for platinum-resistant ovarian cancer, in concordance with liposomal doxorubicin [2, 3]. In two phase III trials, gemcitabine and liposomal doxorubicin showed comparable therapeutic effect with different spectrum of toxicities. Thus, gemcitabine is a potential candidate for combination therapy involving bevacizumab. In a previous Japanese retrospective study, the response rate of combination chemotherapy with gemcitabine plus bevacizumab and gemcitabine monotherapy were 38.9 and 3.4%, respectively. Additionally, PFS and overall survival (OS) of combination chemotherapy with gemcitabine plus bevacizumab were superior [4]. However, there is no prospective study of this combination chemotherapy.

Therefore, we conducted a phase II study to assess the clinical activity and toxicity of combination therapy with gemcitabine and bevacizumab in women with platinum-resistant recurrent epithelial ovarian, primary peritoneal, or fallopian tube cancer.

## Methods

### Patients

Between April 1, 2015 and December 31, 2018, patients with platinum-resistant recurrent epithelial ovarian, primary peritoneal, or fallopian tube cancer were enrolled. Eligible patients were women aged ≥18 years who met the following criteria: (1) histologically confirmed diagnosis of epithelial ovarian, primary peritoneal, or fallopian tube cancer that had progressed within 6 months from completing the last platinum-based chemotherapy (platinum-resistant disease) or progressed during the previous platinum-based chemotherapy (platinum-refractory disease); (2) administration of up to three regimens of chemotherapy; (3) Eastern Cooperative Oncology Group performance status of 0–2; (4) life expectancy of ≥3 months; (5) adequate bone marrow and organ function (neutrophil count, ≥1500 cells/mm^3^; platelet count, ≥100,000/mm^3^; serum transaminase level, up to two times the upper limit of the normal range; total bilirubin level, ≤1.5 mg/dL; and serum creatinine level, ≤1.5 mg/dL); and (6) normal electrocardiography findings.

The article "A phase II study of the combination chemotherapy of bevacizumab and gemcitabine in women with platinum-resistant recurrent epithelial ovarian, primary peritoneal, or fallopian tube cancer" was published in 2020. Journal: J Ovarian Res.

We excluded women with a history of bowel obstruction, abdominal fistula or gastrointestinal (GI) perforation, evidence of rectosigmoid or bowel involvement on computed tomography, clinical symptoms of bowel obstruction. Additional exclusion criteria were prior radiotherapy to the pelvis or abdomen, surgery within 4 weeks before starting the protocol therapy, anticipated need for major surgery during the protocol therapy and a non-healing wound, ulcer, or bone fracture. Moreover, patients with pleural effusion or ascites that required persistent drainage, active concomitant malignancy, or serious concomitant medical illnesses, including uncontrolled infection, uncontrolled hypertension, active clinically significant cardiovascular disease, history or evidence of thrombotic or hemorrhagic disorders within 6 months before the first study treatment, untreated and/or symptomatic central nervous system disease, were considered ineligible.

### Chemotherapy regimen

The treatment protocol included intravenous (IV) infusion of gemcitabine at 1000 mg/m^2^ in 100 mL of saline over a period of 1 h on days 1 and 8, and IV infusion of bevacizumab at 15 mg/kg in 100 mL of saline over a period of 30 min on day 1. At the first cycle, bevacizumab was administered over a period of 90 min. If no infusion reaction occurred, at the second/third cycle and subsequently, bevacizumab was administered over periods of 60 and 30 min, respectively. All patients were administered standard antiemetic and anti-allergic therapies using dexamethasone. Chemotherapy was scheduled to be repeated every 21 days.

Treatment was delayed when the granulocyte count was < 1500/mm^3^, the platelet count was < 100,000/mm^3^, or any non-hematological toxicity, excluding alopecia, malaise, nausea, and constipation, of grade 2 or higher occurred until the severity of symptoms was not higher than grade 1. Treatment delay was allowed for a maximum of 3 weeks. Administration of bevacizumab was skipped when uncontrolled hypertension (systolic blood pressure, > 140 mmHg or diastolic blood pressure, > 90 mmHg) or proteinuria (urine protein-to-creatinine ratio, ≥3.5) was noted. Administration of gemcitabine on day 8 was also delayed up to 3 weeks when an absolute neutrophil count of less than 500 cells/mm^3^ or a platelet count of less than 50,000 /mm^3^.

The gemcitabine dose was reduced to 800 mg/mm^3^ in response to febrile neutropenia, treatment delay by 15–21 days because of prolonged toxicity, or grade 3 non-hematological toxicity. The bevacizumab dose was not reduced for toxicity. Chemotherapy was discontinued in patients experiencing the following: (1) delay in treatment by more than 21 days because of any toxicity; (2) need for greater than level 1 dose reduction of gemcitabine for any toxicity; (3) grade 4 non-hematological toxicity; and (4) disease progression. Additionally, chemotherapy was discontinued in patients who refused treatment.

The article "A phase II study of the combination chemotherapy of bevacizumab and gemcitabine in women with platinum-resistant recurrent epithelial ovarian, primary peritoneal, or fallopian tube cancer" was published in 2020. Journal: J Ovarian Res.

### Evaluation plan

The primary endpoint was the rate of patients who completed ≥3 cycles of the protocol therapy. The secondary endpoints were PFS, OS, the rate of response, and the rate of dose-limiting toxicities, including bowel perforation, febrile neutropenia, and grade 4 thrombocytopenia. In AURELIA trial, patients who completed 3 or more cycles of protocol treatment in monotherapy arm and bevacizumab combination arm were 60 and 85%, respectively [1]. The required sample size was estimated based on a threshold rate of 60% and expected rate of 85, 80% power, and an alpha value of 0.05 (one-sided). The target sample size was determined to be at least 20 patients. The incidence of chemotherapy-induced toxicity was evaluated using a self-reported questionnaire and was graded according to the Common Terminology Criteria for Adverse Events version 4.0. Tumors were evaluated using contrast-enhanced computed tomography every two cycles. The response to chemotherapy was evaluated according to the Response Evaluation Criteria in Solid Tumors 1.1. PFS was defined as the time from patient registration to disease progression, death from any cause, or last contact. OS was defined as the time from patient registration to death from any cause or last contact. PFS and OS were estimated with the Kaplan–Meier method using GraphPad Prism graphing and statistics software (version 7.0a; GraphPad Software, Inc., La Jolla, CA).

### Ethics statement

The study protocol was approved by the local ethics committee of Hyogo Cancer Center before the initiation of patient recruitment, and the study was conducted in accordance with the ethical principles described in the Declaration of Helsinki. All patients provided written informed consent. This study was registered in the University Medical Information Network (UMIN) Clinical Trials Registry (No. 000016619).

## Results

### Patient characteristics

Between April 1, 2015 and December 31, 2018, 20 patients were enrolled into this study. However, one patient declined study treatment after registration. In Japan, a new legislation to regulate clinical research was applicable from April 2019. We have decided to close the new registration to this study by December 31, 2018 in an early stage, because this study have not met the legislation. So, we could not satisfy the planned number of patients. The patient characteristics are presented in Table 1. The median patient age was 57 years (range, 46–75 years). Of the 19 patients, 15 (79%) had a PS of 0 and 4 had a PS of 1. Additionally, 12 patients had high-grade serous carcinoma, 1 had endometrial carcinoma, 4 had clear cell carcinoma, and 2 had other types of histology. Moreover, 14 patients received 1 regimen of platinum-based chemotherapy and five received 2 regimens. Furthermore, 7 patients had platinum-refractory and 12 had platinum-resistant recurrent ovarian cancer.

The article "A phase II study of the combination chemotherapy of bevacizumab and gemcitabine in women with platinum-resistant recurrent epithelial ovarian, primary peritoneal, or fallopian tube cancer" was published in 2020. Journal: J Ovarian Res.

**Table 1:** Patient characteristics

Age, median (range) (years)	57 (46–75)
Performance status, n	
0	15
1	4
≥ 2	0
Histology, n	
High-grade serous	12
Endometrial	1
Clear cell	4
Others	2
Previous platinum-based chemotherapy	
1	14
2	5
Platinum-free interval (months)	
0	7
1–2	1
3–4	5
5	6

### Efficacy

Among the 19 patients, 18 (95%) received ≥3 and 9 (47%) received ≥6 cycles of the study chemotherapy (Table 2). The median number of completed chemotherapy cycles was 4 (range, 1–19 cycles). Three patients were able to continue treatment for > 12 months, and they completed 15, 17, and a maximum of 20 cycles of chemotherapy. The reasons for discontinuation were disease progression in 9 patients, treatment delay beyond 3 weeks because of hematologic toxicity in 3, patient refusal in 2, prolonged grade 3 protein urea in 1, prolonged grade 2 nasal bleeding in 1, pelvic abscess requiring surgical drainage in 1, life-threatening interstitial pneumonia in 1, and life-threatening pulmonary thromboembolism in 1. Three patients needed dose reduction of gemcitabine to 800 mg/m^2^ due to treatment delay by 15 to 21 days on day1. There was no treatment delay more than 14 days on day 8.

**Table 2:** Completed chemotherapy cycles and the reason of discontinuation

Completed cycles	N
1	1
2	0
3	6
4	0
5	3
6	0
7	2
8	1
9	1
10	1
11-	4
Median 5 (1–20)	
Disease progression	9
Delay due to hematologic-toxicity	3
Patient refusal	2
Protein urea	1
Pelvic abscess	1
Interstitial pneumonia	1
Nasal bleeding	1
Pulmonary thromboembolism	1

Among the 19 patients, 8 (42%) showed objective responses (complete response in 3 and partial response in 5) and 8 showed stable disease. The clinical control rate was 84% (16/19 patients). The median PFS duration was 5.1 months, and the median OS duration was 21.3 months (Figs. 1 and 2).

**Fig. 1:** Progression-free survival (PFS) estimated using the Kaplan–Meier method

**Fig. 2:** Overall survival (OS) estimated using the Kaplan–Meier method

The article "A phase II study of the combination chemotherapy of bevacizumab and gemcitabine in women with platinum-resistant recurrent epithelial ovarian, primary peritoneal, or fallopian tube cancer" was published in 2020. Journal: J Ovarian Res.

### Toxicity

Hematological and non-hematological toxicities are presented in Table 3. Hematological toxicities included grade 3 or 4 neutropenia in 9 patients (47%), grade 3 or 4 anemia in 2 (11%), and grade 3 or 4 thrombocytopenia in 1 (5%). No patient received blood transfusion. Grade 3 or more severe non-hematological toxicities included grade 3 aspartate aminotransferase/ alanine aminotransferase increase in two patients, grade 3 hypertension in 1, grade 3 protein urea in 1, life-threatening pulmonary embolism in 1, and interstitial pneumonia in 1. There was no patient encountered GI perforation. Additionally, no treatment-related death was observed.

**Table 3:** Toxicity (*N* = 19)

Event	Grade				
	1	2	3	4	Grade 3/4 (%)
White blood cell decrease	12	2	0	0	0
Neutrophil decrease	3	2	7	2	9 (47)
Febrile neutropenia	–	–	0	0	0
Anemia	8	5	2	0	2 (11)
Platelet count decrease	3	1	1	0	1 (5)
	Grade 2/3/4 (%)				
Nausea	3	2	0	0	2 (11)
Vomiting	1	0	0	0	0
Mucositis oral	2	0	0	0	0
GI perforation	0	0	0	0	0
Sensory neuropathy	3	1	0	0	1 (5)
Motor neuropathy	0	0	0	0	0
Hypertension	7	2	1	0	3 (16)
Protein urea	8	3	1	0	4 (21)
Fatigue	3	0	0	0	0
AST/ALT increase	3	0	2	0	2 (11)
Thromboembolic event	0	0	1	0	1 (5)
Nasal bleeding	0	1	0	0	1 (5)
Interstitial pneumonia	0	0	1	0	1 (5)

Common Terminology Criteria for Adverse Events v4.0

*GI* gastrointestinal, *AST* aspartate aminotransferase, *ALT* alanine aminotransferase

## Discussion

The present study confirmed the feasibility, efficacy and safety of combination chemotherapy with gemcitabine and bevacizumab in women with platinum-resistant recurrent epithelial ovarian, primary peritoneal, or fallopian tube cancer. Among the 19 patients, 18 (95%) received ≥3 cycles of the study chemotherapy, which met the primary endpoint of this study. The completion rate exceeded which of the AURELIA trial [1]. In AURELIA trial, patients who completed 3 or more cycles of protocol treatment in monotherapy arm and bevacizumab combination arm ware 60 and 85%, respectively.

The clinical control rate according to the RECIST was 84% (complete response rate of 16%, partial response rate of 26%, and stable disease rate of 42%) in this study. Additionally, the median PFS duration was 5.1 months, and the median OS duration was 21.3 months. In a previous Japanese retrospective study, the clinical control rate of combination chemotherapy with gemcitabine and bevacizumab was 88.9% (complete response rate of 0%, partial response rate of 38.9%, and stable disease rate of 50%) [4]. Although there was no patient with complete response, the objective response rate and the clinical control rate were comparable with the results of our study. In the AURELIA trial, the overall response rate evaluated according to the RECIST was 27.3% in the bevacizumab combination arm, and the median PFS and OS durations were 6.7 and 16.6 months, respectively [1]. The efficacy of the combination of gemcitabine and bevacizumab appears to be comparable with that of the combination of bevacizumab and another single-agent.

The article "A phase II study of the combination chemotherapy of bevacizumab and gemcitabine in women with platinum-resistant recurrent epithelial ovarian, primary peritoneal, or fallopian tube cancer" was published in 2020. Journal: J Ovarian Res.

In the present study, the spectrum of toxicities of gemcitabine and bevacizumab did not overlap. With gemcitabine and bevacizumab, the grade 3/4 hematologic toxicities were neutropenia in nine patients (47%), anemia in 2 (11%), and thrombocytopenia in 1 (5%). These toxicities were probably related to the administration of gemcitabine. On the other hand, bevacizumab-induced toxicities were grade 3 hypertension in one patient (5%), grade 3 protein urea in 1 (5%), and grade 2 nasal bleeding in 1 (5%). Grade 3 pulmonary thromboembolism in a patient with clear cell carcinoma was believed to be caused by worsening of the primary disease. The causes of grade 3 aspartate aminotransferase/ alanine aminotransferase increase and grade 3 interstitial pneumonia were not clear, although they were believed to be related to gemcitabine or bevacizumab. There was no patient encountered GI perforation. Thus, gemcitabine is believed to be one of the most suitable agents to combine with bevacizumab in terms of toxicity.

The weakness of this study was the absence of an assessment of quality of life (QOL). Nevertheless, QOL during administration of gemcitabine and bevacizumab combination therapy was believed to be good, as refusal to continue chemotherapy was rare. To strengthen the availability of this combination chemotherapy, QOL assessment may be essential in further studies.

Previous studies on colorectal cancer showed prolonged OS in patients who continuously received chemotherapy plus bevacizumab beyond disease progression from first- to second-line therapy compared with those who received chemotherapy alone [5, 6]. Similarly, prolonged PFS was shown in breast cancer patients who received chemotherapy plus bevacizumab beyond progression disease compared with chemotherapy alone [7]. The Japanese Gynecologic Oncology Group is currently performing a phase II study to confirm the hypothesis that PFS is better in patients treated with a combination of single-agent chemotherapy and bevacizumab than in those treated with single-agent chemotherapy alone in the setting beyond progression disease following prior bevacizumab treatment [8]. Recently, a study reported stable disease for 29 months in a patient with platinum-resistant recurrent ovarian cancer who received gemcitabine and bevacizumab combination chemotherapy [9]. This patient had received bevacizumab maintenance therapy. Combination chemotherapy with gemcitabine and bevacizumab might be effective in the setting beyond disease progression. However, we did not include patients with previous bevacizumab administration in this study.

The article "A phase II study of the combination chemotherapy of bevacizumab and gemcitabine in women with platinum-resistant recurrent epithelial ovarian, primary peritoneal, or fallopian tube cancer" was published in 2020. Journal: J Ovarian Res.

In conclusion, combination chemotherapy with gemcitabine and bevacizumab was feasible, effective and safe in women with platinum-resistant recurrent epithelial ovarian, primary peritoneal, or fallopian tube cancer. This combination chemotherapy may be explored in a further randomized trial.

## Data Availability

All data are available from the corresponding author on reasonable requests.
